# Prostaglandin E_2_ Signals Through E Prostanoid Receptor 2 to Inhibit Mitochondrial Superoxide Formation and the Ensuing Downstream Cytotoxic and Genotoxic Effects Induced by Arsenite

**DOI:** 10.3389/fphar.2019.00781

**Published:** 2019-07-12

**Authors:** Liana Cerioni, Andrea Guidarelli, Mara Fiorani, Orazio Cantoni

**Affiliations:** Department of Biomolecular Sciences, University of Urbino Carlo Bo, Urbino, Italy

**Keywords:** PGE_2_, arsenite, mitoO_2_^−.^, MPT, cytotoxicity, genotoxicity

## Abstract

We investigated the effects of prostaglandin E_2_ (PGE_2_), an important inflammatory lipid mediator, on the cytotoxicity–genotoxicity induced by arsenite. With the use of a toxicity paradigm in which the metalloid uniquely induces mitochondrial superoxide (mitoO_2_^−.^) formation, PGE_2_ promoted conditions favoring the cytosolic accumulation of Bad and Bax and abolished mitochondrial permeability transition (MPT) and the ensuing lethal response through an E prostanoid receptor 2/adenylyl cyclase/protein kinase A (PKA) dependent signaling. It was, however, interesting to observe that, under the same conditions, PGE_2_ also abolished the DNA-damaging effects of arsenite and that this response was associated with an unexpected suppression of mitoO_2_^−.^ formation. We conclude that PGE_2_ promotes PKA-dependent inhibition of mitoO_2_^−.^ formation, thereby blunting the downstream responses mediated by these species, leading to DNA strand scission and MPT-dependent apoptosis. These findings are therefore consistent with the possibility that, in cells responding to arsenite with mitoO_2_^−.^ formation, PGE_2_ fails to enhance—but rather decreases—the risk of neoplastic transformation associated with genotoxic events.

## Introduction

Arsenite is a widely distributed environmental toxicant causing an increased incidence of various pathologies and forms of cancer in numerous parts of the planet (Flora, 2011; Shakoor et al., 2017; Minatel et al., 2018). Animal and cell culture studies have demonstrated that the metalloid promotes several critical events, as disturbed Ca^2+^ homeostasis (Banerjee et al., 2011; Suriyo et al., 2012), mitochondrial dysfunction (Flora, 2011; Minatel et al., 2018), autophagy, and apoptosis (Guidarelli et al., 2016a; Guidarelli et al., 2016b). Furthermore, common hallmarks of arsenite toxicity are represented by the formation of mitochondrial (Guidarelli et al., 2016a) and/or NADPH oxidase (Smith et al., 2001; Guidarelli et al., 2016b) and derived superoxide (O_2_^−.^), as well as by the resulting induction of a variety of lesions in different biomolecules (Flora, 2011; Minatel et al., 2018).

We have recently focused our attention on arsenite toxicity using U937 cells, in which exposure to a 2.5 µM concentration of the metalloid selectively promotes a slow and progressive formation of mitochondrial O_2_^−.^ (mitoO_2_^−.^) (Guidarelli et al., 2016a; Guidarelli et al., 2017; Fiorani et al., 2018). This response is preceded by an initial weak activation of the inositol trisphosphate receptor and a subsequent stimulation of the inositol trisphosphate receptor–ryanodine receptor intraluminal crosstalk promoting a large release of the cation from the ryanodine receptor to the cytosol (Guidarelli et al., 2018). These conditions were then associated with a remarkable accumulation of the cation in the mitochondria, an event critical for mitoO_2_^−.^ formation (Guidarelli et al., 2019). In addition, mitoO_2_^−.^ was identified as the critical upstream species indirectly responsible, i.e., through the intermediate formation of H_2_O_2_, for the triggering of events associated with vicinal effects culminating in mitochondrial dysfunction/permeability transition (MPT) (Guidarelli et al., 2016a; Fiorani et al., 2018), as well as distal effects, which include the formation of lesions at the level of genomic DNA (Guidarelli et al., 2017). All these effects were then followed by a delayed (i.e., after 24–48 h) apoptotic response, however restricted to a small proportion of cells (Guidarelli et al., 2016a; Guidarelli et al., 2016b; Guidarelli et al., 2017).

The genotoxic response detected under these conditions therefore takes place in a large proportion of the cells exposed to the metalloid, whereas only a small fraction of the same cells is eventually engaged in the apoptotic process (Guidarelli et al., 2016a; Guidarelli et al., 2016b; Guidarelli et al., 2017). In this perspective, the specific treatment paradigm employed in these studies appears relevant for addressing questions related to arsenite genotoxicity. It is indeed reasonable to expect an increased risk of neoplastic transformation in viable cells concurrently accumulating a genotoxic damage. Obviously, the risk would be even more augmented in cells concomitantly exposed to arsenite and additional agents promoting cytoprotection.

It is well established that the process of carcinogenesis is often associated with inflammation and that this condition, by enhancing the formation/expression of both toxic and cytoprotective molecules, is in turn involved in the regulation of the initiation and promotion phases of carcinogenesis (Aggarwal et al., 2006; Sethi et al., 2012). As an example, the inflammatory process is associated with the expression of diverse NF-kB-dependent genes (Tak and Firestein, 2001), which include the one encoding for inducible cyclooxygenase-2, an enzyme responsible for the formation of very large amounts of prostaglandins, as prostaglandin E_2_ (PGE_2_).

PGE_2_, an important inflammatory lipid mediator, is involved in the regulation of an array of physiological as well as pathological activities (Gomez et al., 2013; Wang et al., 2018). In particular, once secreted by inflammatory cells, PGE_2_ acts in an autocrine or paracrine manner on four different E prostanoid (EP) receptors. EP_1_ signals through Gq proteins to elevate Ca^2+^, EP_2_ and EP_4_ through Gs proteins to activate adenylyl cyclase, and EP_3_ through Gi proteins to decrease adenylyl cyclase activity (Markovic et al., 2017).

PGE_2_ mediates cytoprotection in various conditions (Vassiliou et al., 2004; Kamiyama et al., 2006; Leone et al., 2007; Ghosh et al., 2010; Shehzad et al., 2016) and has been implicated in other processes associated with carcinogenesis (Kuwano et al., 2004; Ghosh et al., 2010; Roberts et al., 2011). Numerous tumors indeed display enhanced cyclooxygenase-2 expression (Sano et al., 1995; Liu and Rose, 1996; Huang et al., 1998; Ghosh et al., 2010; Rundhaug et al., 2011), and inhibition of cyclooxygenase-2 activity has been associated with a decreased risk of carcinogenesis (Arun and Goss, 2004; Ghosh et al., 2010; Liu et al., 2015; Guarnieri, 2016).

Various studies have recently proposed that PGE_2_ may play an important role through the EP_2_ receptor signaling, associated with increased cyclic adenosine monophosphate (cAMP) levels and stimulation of protein kinase A (PKA) activity, reported to phosphorylate various critical targets implicated in the induction of tumor cell survival (Yang et al., 2005; Loh et al., 2015; Whiting et al., 2015).

Based on the above considerations, we decided to address the question of whether PGE_2_ promotes effects on the cytotoxic and genotoxic responses mediated by arsenite. For this purpose, we used the same U937 cell line previously employed to carefully define conditions in which the metalloid selectively stimulates mitoO_2_^−.^ formation (Guidarelli et al., 2016a) and the ensuing MPT-dependent apoptosis (Guidarelli et al., 2016a; Guidarelli et al., 2017; Fiorani et al., 2018), as well as the strand scission of genomic DNA (Guidarelli et al., 2017). An additional important feature of U937 cells is related to the expression of EP_2_ receptors coupled to a PKA-dependent survival signaling leading to Bad phosphorylation (Tommasini et al., 2008).

We report that PGE_2_ abolishes arsenite toxicity through an EP_2_ receptor/PKA dependent signaling. Under these conditions, an increased Bad phosphorylation on serine 112 (Ser^112^) associated with the cytosolic accumulation of the protein was readily detected and linked to prevention of Bax translocation and MPT. It was, however, interesting to observe that these cytoprotective effects were associated with the parallel prevention of DNA strand scission, an event mediated by an unexpected suppression of mitoO_2_^−.^ formation. It therefore appears that PGE_2_ signals affect a specific target involved in mitoO_2_^−.^ formation and hence prevents all the downstream responses mediated by these species, which include MPT-dependent apoptosis and DNA single-strand breakage.

## Materials and Methods

### Chemicals

Sodium arsenite, PGE_2_, butaprost, AH6809, AH23848, KT5720, forskolin, 3-isobutyl-1-methylxanthine (IBMX), rotenone, catalase, 3-amino-1,2,4,-triazole (ATZ), Hoechst 33342, and most of the reagent-grade chemicals were purchased from Sigma-Aldrich (Milan, Italy). Cyclosporin A (CsA) was from Novartis (Bern, Switzerland). Dihydrorhodamine 123 (DHR), MitoSOX red, and MitoTracker Red CMXRos were purchased from Molecular Probes (Leiden, The Netherlands).

### Antibodies

The antibodies against cytochrome *c*, actin, and HSP-60 as well as the horseradish peroxidase-conjugated secondary antibody were purchased from Santa Cruz Biotechnology (Santa Cruz, CA). Bad and Bax antibodies were from BD Transduction Laboratories (Lexington, KY). The antibody recognizing Bad phosphorylated at Ser^112^ was from Cell Signaling Technology (Beverly, MA).

### Cell Culture and Treatment Conditions

U937 human myeloid leukemia cells were cultured in suspension in RPMI 1640 medium (Sigma-Aldrich). Culture media were supplemented with 10% fetal bovine serum (EuroClone, Celbio Biotecnologie, Milan, Italy), penicillin (100 U/ml), and streptomycin (100 mg/ml) (EuroClone). Cells were grown at 37°C in T-75 tissue culture flasks (Corning Inc., Corning, NY) gassed with an atmosphere of 95% air–5% CO_2_. Sodium arsenite was prepared as a 1 mM stock solution in saline A (140 mM NaCl, 5 mM KCl, 4 mM NaHCO_3_, and 5 mM glucose; pH 7.4) and stored at 4°C. Cells (1 × 10^5^ cells/ml) were exposed to arsenite in complete RPMI 1640 culture medium, as reported in the legends to the figures. In experiments involving catalase depletion, the cells (5 × 10^6^/20 ml) were incubated for 6 h at 37°C in Roswell Memorial Park Institute (RMPI) medium containing 10 mM ATZ, an irreversible inhibitor of catalase (Darr and Fridovich, 1986). PGE_2_, butaprost, rotenone, catalase, or CsA were given to the culture 5 min prior to arsenite. AH6809, AH23848, KT5720, forskolin, and IBMX were added to the culture 30 min prior to arsenite.

### Measurement of Mitochondrial Membrane Potential

The cells were incubated for 30 min with 50 nM MitoTracker Red CMXRos prior to the end of the incubation with arsenite. After treatments, the cells were washed three times, and fluorescence images were captured with a BX-51 microscope (Olympus, Milan, Italy), equipped with a SPOT-RT camera unit (Diagnostic Instruments, Delta Sistemi, Rome, Italy) using an Olympus LCAch 40×/0.55 objective lens. The excitation and emission wavelengths were 545 and 610 nm, respectively, with a 5-nm slit width for both emission and excitation. Images were collected with exposure times of 100–400 ms, digitally acquired and processed for fluorescence determination at the single cell level on a personal computer using Scion Image software (Scion Corp., Frederick, MD). Mean fluorescence values were determined by averaging the fluorescence values of at least 50 cells/treatment condition/experiment.

### Sub-Cellular Fractionation and Western Blot Analysis

After treatments, the cells were processed to obtain the mitochondrial fractions, as described in Cantoni et al. (2008), and the whole cell lysates, as described in Guidarelli et al. (2005). Equal amounts of proteins (25 µg) were loaded in each lane, separated by polyacrylamide gel electrophoresis in the presence of sodium dodecyl sulfate, transferred to polyvinylidene difluoride membranes, and probed with antibodies against cytochrome *c*, Bad, Bax, Bad phosphorylated at Ser^112^, HSP-60, or actin. Details on Western blotting apparatus and conditions are reported elsewhere (Cantoni et al., 2008). Antibodies against actin and HSP-60 were used to assess the equal loading of the lanes and the purity of the fractions. Relative amounts of proteins were quantified by densitometric analysis using Image J software.

### Fluorogenic Caspase 3 Assay

Caspase 3-like activity was monitored as described in Guidarelli et al. (2005). Briefly, the cells were lysed, and aliquots of the extract (30 mg proteins) were incubated with 12 µM Ac-DEVD-AMC, at 30°C. Caspase 3-like activity was determined fluorometrically (excitation at 360 nm and emission at 460 nm) by quantifying the release of aminomethyl coumarin (AMC) from cleaved caspase 3 substrate (Ac-DEVD-AMC).

### Cytotoxicity Assay

Cytotoxicity was determined with the trypan blue exclusion assay. Briefly, an aliquot of the cell suspension was diluted 1:1 (v/v) with 0.4% trypan blue, and the viable cells (i.e., those excluding trypan blue) were counted with a hemocytometer.

### Analysis of Apoptosis with Hoechst 33342 Assay

After treatments, the cells were incubated for 5 min with 10 μM Hoechst 33342 and then analyzed with a fluorescence microscope to assess their nuclear morphology (chromatin condensation and fragmentation). Cells with homogeneously stained nuclei were considered viable.

### Measurement of DNA Single-Strand Breakage by the Alkaline Halo Assay

DNA single-strand breakage was determined using the alkaline halo assay developed in our laboratory (Cantoni and Guidarelli, 2008). It is important to note that, although we refer to DNA strand scission throughout the text, the DNA nicks measured by this technique under alkaline conditions may in fact include alkali labile sites in addition to direct strand breaks. Details on the alkaline halo assay and processing of fluorescence images and on the calculation of the experimental results are also given in Cantoni and Guidarelli (2008). DNA single-strand breakage was quantified by calculating the nuclear spreading factor value, representing the ratio between the area of the halo (obtained by subtracting the area of the nucleus from the total area, nucleus + halo) and that of the nucleus, from 50 to 75 randomly selected cells/experiment/treatment condition.

### DHR and MitoSOX Red Fluorescence Assays

The cells were supplemented with either 10 µM DHR or 5 µM MitoSOX red, 30 min prior to the end of the treatments, washed three times with saline A, and subsequently analyzed with a fluorescence microscope. The resulting images were taken and processed as described above. The excitation and emission wavelengths were 488 and 515 nm (DHR) and 510 and 580 nm (MitoSOX red), with a 5-nm slit width for both emission and excitation. Mean fluorescence values were determined by averaging the fluorescence values of at least 50 cells/treatment condition/experiment.

### Aconitase Activity

After treatments, the cells were washed twice with saline A, re-suspended in lysis buffer (50 mM Tris–HCl, 2 mM Na-citrate, and 0.6 mM MnCl_2_, pH 7.4), and finally sonicated three times on ice by using the Sonicator Ultrasonic Liquid Processor XL (Heat System-Ultrasonics, Inc., NY) operating at 20 W (30 s). The resulting homogenates were centrifuged for 5 min at 18,000 ×g at 4°C. Aconitase activity was determined spectrophotometrically in the supernatants at 340 nm, as described in Gardner (2002).

### Statistical Analysis

The results are expressed as means ± SD. Statistical differences were analyzed by one-way ANOVA followed by Dunnett’s test for multiple comparison or two-way ANOVA followed by Bonferroni’s test for multiple comparison. A value of *p* < 0.05 was considered significant.

## Results

### Cytoprotection Mediated by PGE_2_ Supplementation: Involvement of EP_2_ Receptors

A 16-h exposure of U937 cells to 2.5 µM arsenite promotes a decline in mitochondrial membrane potential sensitive to 0.5 µM CsA supplementation (**Figure 1A**). Interestingly, PGE_2_ (3 µM) mimicked the protective effects mediated by the MPT inhibitor. The concentration dependence of the inhibitory effects mediated by PGE_2_ is illustrated in **Figure 1B**.

**Figure 1:** Prostaglandin E_2_ (PGE_2_) prevents the deleterious effects of arsenite on mitochondrial function and integrity *via* a mechanism involving EP_2_-receptor stimulation and downstream activation of protein kinase A (PKA). **(A)** Cells were exposed for 16 h to 2.5 µM arsenite in the absence or presence of PGE_2_ (3 µM), or cyclosporin A (CsA) (0.5 µM), and then processed for the assessment of the mitochondrial membrane potential. **(B)** Cells were exposed to arsenite in the absence or presence of increasing concentrations of PGE_2_ and then processed as indicated in A. **(C)** Cells were exposed to arsenite in the absence or presence of PGE_2_, butaprost (50 µM), 3-isobutyl-1-methylxanthine (IBMX) (300 µM), forskolin (50 µM), AH6809 (50 µM), AH23848 (50 µM), and KT5720 (3 µM), alone or in combination, as indicated in the figure. After treatments, the cells were processed for the assessment of the mitochondrial membrane potential. In other experiments, the cells were treated as indicated in C and then processed to purify the mitochondrial fraction for Western blot analysis of cytochrome *c* (cyt c) **(D, E)**. Blots, representative of three separate experiments with similar outcomes, were also probed for actin and HSP-60. Results represent the means ± SD calculated from at least three separate experiments. *p < 0.01 as compared with untreated cells. (*)*p* < 0.01; as compared with cells treated with arsenite (**A, C–E**, one-way ANOVA followed by Dunnett’s test; **B**, two-way ANOVA followed by Bonferroni’s test).

As indicated in **Figure 1C**, the protective effects of PGE_2_ were abolished by AH6809 (50 µM), an EP_2_ antagonist (Markovic et al., 2017), with hardly any effect detected with the EP_4_ receptor antagonist AH23848 (50 µM) (Markovic et al., 2017). Furthermore, butaprost, an EP_2_ receptor agonist (Markovic et al., 2017), mimicked the protective effects of PGE_2_ with an identical specific sensitivity to AH6809. Sulprostone (50 µM), an EP_1_–EP_3_ receptor agonist (Markovic et al., 2017), failed to recapitulate the effects mediated by PGE_2_ (not shown). Finally AH6809, or AH23848, produced hardly any effect in cells exposed to arsenite alone, or in the absence of additional treatments. PGE_2_, or butaprost, also failed to produce effects in the absence of additional treatments.

The CsA-sensitive loss of mitochondrial membrane potential induced by arsenite is associated with a CsA-sensitive release of cytochrome *c* (**Figure 1D**) and followed (48 h) by CsA-sensitive activation of caspase 3 (**Figure 2A**), reduction in viable cell counts (**Figure 2B**), and increased apoptosis (**Figure 2C**). All these events were prevented by PGE_2_, or butaprost, once again *via* mechanisms sensitive to AH6809 and insensitive to AH23848.

**Figure 2:** PGE_2_ prevents the apoptotic response mediated by arsenite *via* a mechanism involving EP_2_-receptor stimulation and downstream activation of PKA. **(A–C)** Cells were treated as indicated in the figure and using the same conditions detailed in the legend to **Figure 1C–E**. After 48 h, the cells were processed for the assessment of caspase 3 activity **(A)** and toxicity by either quantifying the number of viable cells **(B)** or measuring the percentage of apoptotic cells, i.e., cells displaying chromatin fragmentation/condensation **(C)**. Results represent the means ± SD calculated from at least three separate experiments. *p < 0.01, as compared with untreated cells (one-way ANOVA followed by Dunnett’s test).

These results indicate that PGE_2_ prevents the dissipation of mitochondrial membrane potential and the downstream triggering of the apoptotic cascade mediated by arsenite by signaling *via* EP_2_ receptors.

### Cytoprotection Mediated by PGE_2_ Supplementation: Involvement of PKA

The EP_2_ receptor signaling leads to adenylyl cyclase activation and increased cAMP formation (Markovic et al., 2017). The involvement of these receptors in the above protective effects is therefore further established by the observation that the protective effects of PGE_2_ on the arsenite-induced inhibition of mitochondrial membrane potential (**Figure 1C**), mitochondrial loss of cytochrome *c* (**Figure 1E**), caspase 3 activation (**Figure 2A**), decreased cell counts (**Figure 2B**), and increased apoptosis (**Figure 2C**) are mimicked by the phosphodiesterase inhibitor IBMX (300 µM) or the adenylyl cyclase activator forskolin (50 µM) (Dessauer et al., 2017). Of note, the observed protective effects were sensitive to the PKA inhibitor KT5720 (3 µM) (Murray, 2008), regardless of whether mediated by PGE_2_, butaprost, IBMX, or forskolin (**Figure 1C–E** and **Figure 2A–C**). AH6809 instead failed to prevent the protective responses mediated by IBMX and forskolin, thereby providing an indication for the specificity of its effects as an EP_2_ receptor antagonist. Finally IBMX, or forskolin, produced hardly any effect in the absence of additional treatments.

Collectively, the results illustrated in this section provide compelling evidence for the involvement of PKA in the EP_2_-mediated PGE_2_ signaling leading to inhibition of mitochondrial dysfunction and cytotoxicity induced by arsenite.

### Prevention of the Arsenite-Dependent Mitochondrial Dysfunction by PGE_2_ Is Associated With Inhibition of the Mitochondrial Translocation of Bad and Bax

The protective effects mediated by PGE_2_ in cells exposed to arsenite are upstream to MPT. In principle, a potential target for PKA in this signaling is represented by Bad, which may translocate to mitochondria and heterodimerize with Bcl-2 and/or Bcl-X_L_, thereby hampering their ability to prevent MPT (Correia et al., 2015; Doerflinger et al., 2015; Edlich, 2018). PKA-dependent phosphorylation on Ser^112^ is indeed reported to enforce the cytosolic localization of Bad, thereby preventing its translocation to mitochondria and the ensuing MPT (Yang et al., 2005; Danial, 2008).

The results illustrated in **Figure 3A** indicate that a 16-h exposure to the metalloid promotes the mitochondrial translocation of Bad and that this event is insensitive to KT5720. Furthermore, the mitochondrial accumulation of Bad was prevented by PGE_2_, or forskolin, *via* KT5720-sensitive mechanisms. Arsenite also caused a decrease in Ser^112^ phosphorylation, and this event was inhibited by PGE_2_ or forskolin, once again *via* a mechanism sensitive to KT5720 (**Figure 3B**).

**Figure 3:** PGE_2_ prevents the mitochondrial translocation of Bad and Bax induced by arsenite. Cells received the treatments indicated in the figure prior to the addition of arsenite. After 16 h, the cells were processed to obtain the mitochondrial fraction for Western blot analysis using anti-Bad **(A)** and anti-Bax **(C)** antibodies. In other experiments, the cells were treated as indicated above and lysed prior to Western blot analysis using an antibody recognizing Bad phosphorylated at Ser^112^ **(B)**. Blots shown are also probed for actin, or HSP-60, and are representative of three separate experiments with similar outcomes. *p < 0.01, as compared with untreated cells (one-way ANOVA followed by Dunnett’s test).

We finally performed experiments showing that arsenite also induces the mitochondrial translocation of Bax and that this event is inhibited by PGE_2_ through a KT5720-sensitive mechanism (**Figure 3C**).

These results indicate that arsenite promotes the mitochondrial translocation of Bad and Bax and are consistent with the possibility that Bad represents the target of the PGE_2_/PKA-dependent signaling.

### PGE_2_ Prevents Mitochondrial Superoxide Formation and the Ensuing Intra-Mitochondrial and Extra-Mitochondrial Effects Induced by Arsenite

Having established that PGE_2_ promotes survival in cells exposed to genotoxic levels of arsenite, we wondered whether this lipid mediator also produced effects on the DNA single-strand breakage that, as determined in our previous studies (Guidarelli et al., 2017), results from two separate mechanisms. The first one is mediated by the conversion of mitochondrial O_2_^−.^ to H_2_O_2_, which can now exit the mitochondria, diffuse, and eventually produce effects in distal targets, as the DNA. The second mechanism is instead associated with the onset of MPT, and the ensuing triggering of events apparently enforcing the mitochondrial formation of H_2_O_2_.

Consistent with our previous findings (Guidarelli et al., 2017), the alkaline halo assay revealed that a 16-h exposure to arsenite promotes DNA strand scission in most of the cells (not shown) and that this response is partially reduced by the MPT inhibitor CsA and instead abolished by enzymatically active catalase, with hardly any effect detected with the boiled enzyme (**Figure 4A**). In addition, the DNA-damaging response was significantly enhanced by ATZ under conditions in which catalase activity was significantly reduced (about 70%, not shown) (Guidarelli et al., 1997). We also report that the effects of catalase are mimicked by rotenone, an inhibitor of complex I (Degli Esposti, 1998) preventing mitoO_2_^−.^ formation induced by arsenite (Guidarelli et al., 2016a), and that KT5720 fails to affect the DNA-damaging response induced by arsenite alone (not shown) or combined with any of the above treatments (**Figure 4A**).

**Figure 4:** PGE_2_ prevents the formation of mitoO_2_^−.^ induced by arsenite and the ensuing mitochondrial and extramitochondrial effects. Cells were exposed for 16 h to arsenite, in the absence or presence of CsA, enzymatically active or heat-inactivated catalase (50 U/ml), rotenone (0.5 µM), PGE_2_, IBMX, forskolin, or KT5720, as indicated in the figures. In other experiments, the cells were incubated for 6 h with 10 mM 3-amino-1,2,4,-triazole (ATZ) and subsequently treated with arsenite. After treatments, the cells were analyzed for DNA damage **(A)**, dihydrorhodamine 123 (DHR_ fluorescence **(B)**, MitoSOX red fluorescence **(C)**, and aconitase activity **(D)**. Results represent the means ± SD calculated from at least three separate experiments. *p < 0.05; **p < 0.01, as compared with untreated cells (one-way ANOVA followed by Dunnett’s test).

It was very interesting to observe that PGE_2_, IBMX, or forskolin also suppress the DNA damaging response induced by arsenite and that these protective effects, unlike those mediated by catalase or rotenone, are abolished by KT5720 (**Figure 4A**).

These results indicate that the mechanism whereby PGE_2_ inhibits the genotoxic effects of arsenite is specifically linked to the triggering of the PKA signaling, thereby implying that Bad is not a direct target for cytoprotection. Our findings imply the involvement of earlier effects, likely associated with inhibition of mitoO_2_^−.^ formation.

We therefore decided to perform additional studies using two different fluorescence probes, DHR (**Figure 4B**), detecting various reactive species in mitochondrial and extramitochondrial compartments (Gomes et al., 2005), and MitoSOX red (**Figure 4C**), commonly employed to detect mitoO_2_^−.^ in live cells (Mukhopadhyay et al., 2007). The results obtained in these experiments indicated that the resulting fluorescence responses are inhibited by rotenone, as well as PGE_2_, IBMX, or forskolin, with a sensitivity to KT5720 restricted to the last three treatments.

We then moved to other studies measuring the activity of aconitase (**Figure 4D**), a O_2_^−.^-sensitive mitochondrial enzyme (Gardner, 2002). The outcome of these experiments was in line with the above findings, thereby providing further evidence for the specific ability of PGE_2_ to prevent mitoO_2_^−.^ formation *via* a KT5720-sensitive mechanism.

These results therefore indicate that the PGE_2_/PKA-dependent signaling selectively blunts mitoO_2_^−.^/H_2_O_2_ formation elicited by arsenite, thereby preventing the intra-mitochondrial and extra-mitochondrial effects mediated by these radical species.

## Discussion

The present study was undertaken to determine the effects of PGE_2_ on arsenite cytotoxicity–genotoxicity, with the purpose of identifying responses with a potential impact on the carcinogenicity of the metalloid. PGE_2_ indeed promotes cytoprotection in various cellular systems and conditions (Vassiliou et al., 2004; Kamiyama et al., 2006; Leone et al., 2007; Ghosh et al., 2010; Shehzad et al., 2016), and the occurrence of this event in response to the metalloid may favor cellular transformation, in particular if the survival response is paralleled by enhanced or even unaltered formation of arsenite-derived genotoxic species.

We therefore designed our study to determine whether PGE_2_ mediates cytoprotection in a well-established toxicity paradigm in which a low concentration of the metalloid promotes the time-dependent formation of mitoO_2_^−.^, responsible for the triggering of events leading to DNA strand scission in most of the cells (Guidarelli et al., 2017), and to mitochondrial dysfunction/MPT, followed by delayed apoptotic death in a small proportion of the cells (Guidarelli et al., 2016a; Guidarelli et al., 2016b).

We found that, in this toxicity paradigm, PGE_2_ dose dependently inhibits the effects of arsenite on mitochondrial function and integrity (detected as decline of mitochondrial membrane potential and mitochondrial loss of cytochrome *c*) as well as the ensuing downstream events leading to cell death (detected as activation of caspase 3, decreased number of viable cells, and apoptotic chromatin fragmentation).

We then established that the protective effects are mediated by PGE_2_ binding to EP_2_ receptors. This notion is based on the observations that cytoprotection was sensitive to AH6809, an EP_2_ receptor antagonist, and insensitive to the EP_4_ receptor antagonist AH23848. Furthermore butaprost, an EP_2_ receptor agonist, unlike sulprostone, an EP_1_–EP_3_ receptor agonist, recapitulated the effects mediated by PGE_2_ *via* AH6809-sensitive and AH23848-insensitive mechanisms.

A third relevant information is that the protective effects of PGE_2_ were mimicked by the phosphodiesterase inhibitor IBMX, or the adenylyl cyclase activator forskolin, however, through a mechanism insensitive to AH6809. These results are therefore indicative of an involvement of the cAMP signaling and further emphasize the specificity of the effects of AH6809 as an EP_2_ receptor antagonist.

Finally, we provided evidence for an involvement of PKA in the above signaling, as KT5720 suppressed the protective effects of PGE_2_, or butaprost, as well as those mediated by IBMX or forskolin.

The results thus far discussed therefore indicate that PGE_2_ dose dependently prevents the effects of arsenite on the induction of MPT, and the ensuing downstream events leading to apoptosis, by signaling through the EP_2_ receptor/adenylyl cyclase/PKA axis. The concentrations of PGE_2_ resulting in cytoprotection were therefore conditioned by the specific density of the EP_2_ receptors in the U937 cell line used in our experiments.

The PKA signaling potentially activates multiple cytoprotective pathways associated with the suppression of mitochondrial dysfunction and apoptosis (Yang et al., 2005; Loh et al., 2015; Whiting et al., 2015). Among these, a good candidate target is represented by Bad, which may be phosphorylated by PKA on Ser^112^ to enforce its cytosolic localization and mitochondrial translocation (Yang et al., 2005; Danial, 2008). These conditions are associated with the heterodimerization of Bad with other members of the Bcl_2_ family, as Bcl_2_ itself or Bcl-X_L_, thereby hampering their anti-MPT function (Danial, 2008; Correia et al., 2015; Doerflinger et al., 2015; Edlich, 2018). Furthermore, the mitochondrial translocation of Bad is promptly followed by the translocation of Bax, another member of the Bcl_2_ family (Tafani et al., 2001; Cantoni et al., 2008; Doerflinger et al., 2015; Edlich, 2018), which may also heterodimerize with Bcl_2_ or Bcl-X_L_ and hence further reduce their anti-MPT function. In addition, Bax directly causes (Kumarswamy and Chandna, 2009; Correia et al., 2015; Uren et al., 2017), or participates in events causing (Kumarswamy and Chandna, 2009; Raemy and Martinou, 2014), MPT.

Our results showing that arsenite increases the fractions of Bad and Bax associated with the mitochondria are therefore consistent with the possibility that the cytoprotective effects of PGE_2_ are mediated by PKA-dependent phosphorylation of Bad on Ser^112^. This notion was then experimentally established by showing that the mitochondrial translocation of Bad and Bax is inhibited by PGE_2_ *via* a KT5720-sensitive mechanism. Furthermore, the effects of PGE_2_ on both the mitochondrial translocation Bad and its phosphorylation on Ser^112^ were recapitulated by forskolin, once again *via* a KT5720-sensitive mechanism.

The above findings are therefore consistent with the possibility that the effects of PGE_2_ on the EP_2_ receptor/adenylyl cyclase/PKA axis finally lead to Bad phosphorylation-dependent cytoprotection. It is, however, important to note that this conclusion is based on the detection of events taking place 16 h after addition of arsenite, a time at which MPT is detectable in the absence of obvious signs of cell death (Guidarelli et al., 2016a; Guidarelli et al., 2016b). This means that PGE_2_, added to the cultures in parallel with arsenite, may signal and produce early effects, even prior to the specific triggering of events leading to Bad/Bax translocation and induction of MPT. Furthermore, G-protein-coupled receptors rapidly respond to agonist stimulation.

Based on these considerations, the possibility that the above signaling responses are conditioned by earlier effects mediated by PGE_2_ through the PKA-dependent mechanism appears likely. The results from genotoxicity studies put even more weight on this possibility.

This part of the study was preceded by preliminary experiments recapitulating our previous findings indicating that H_2_O_2_, generated upon dismutation of mitoO_2_^−.^, is entirely responsible for the DNA damage induced by the metalloid (Guidarelli et al., 2017). We also reported that part of the mitoO_2_^−.^ is CsA sensitive and hence generated through an MPT-dependent mechanism (Guidarelli et al., 2017). The involvement of H_2_O_2_ was therefore confirmed by showing that the DNA-damaging response is suppressed by enzymatically active catalase and that inhibition of catalase activity is accompanied by the formation of more DNA single strand breaks. In addition, rotenone, which prevents mitoO_2_^−.^ formation and hence the formation of H_2_O_2_, was as effective as catalase in preventing the genotoxic response mediated by arsenite.

In this study, we present the intriguing finding that similar protective effects are induced by PGE_2_, IBMX, or forskolin, which implies the involvement of the same mechanisms previously described in detail in the first part of the study. This notion was more clearly established by showing that KT5720 selectively prevents these protective effects, with hardly any response detected in cells supplemented with rotenone, catalase, or ATZ. These observations are therefore in keeping with the notion that KT5720 exerts its effects *via* selective inhibition of PKA activity and demonstrate that suppression of the DNA damaging response is entirely mediated by activation of the PGE_2_/EP_2_ receptor/adenylyl cyclase/PKA axis.

Based on these findings, two different mechanisms may explain the protective effects of PGE_2_ on arsenite-induced cytotoxicity–genotoxicity: the first one involves inhibition of MPT, and the second, inhibition of mitoO_2_^−.^ formation.

It was then interesting to find that the PKA-sensitive target recruited by PGE_2_ directly blunts mitoO_2_^−^ formation, a notion established using a general probe, DHR, which detects various reactive species, as well as the more specific MitoSOX red, which only allows the detection of mitoO_2_^−.^ Furthermore, an identical outcome was obtained from experiments measuring the activity of aconitase, a mitochondrial O_2_^−.^-sensitive enzyme. These experiments reproducibly demonstrated that PGE_2_ suppresses mitoO_2_^−.^ formation, that the same response is mediated by IBMX or forskolin, and that these protective effects are always sensitive to KT5720.

In conclusion, the present study underscores a novel effect mediated by PGE_2_ in a specific toxicity paradigm involving exposure of U937 cells to a low concentration of arsenite resulting in mitoO_2_^−.^ formation and in the downstream formation of DNA lesions and apoptosis. The novel effect of PGE_2_ was mediated by the activation of the EP_2_/adenylyl cyclase/PKA signaling pathway and was surprisingly associated with the suppression of mitoO_2_^−.^ formation, with an ensuing inhibition of the cytotoxic and genotoxic effects of the metalloid. Despite the limitations of this cell line as a target for arsenite toxicity, we believe that our findings are nevertheless of biological relevance for understanding the effects of the metalloid in various cells types in which it mediates similar upstream responses and triggers the same mechanisms of mitoO_2_^−.^ formation.

Future studies will address the molecular bases of this protective response and investigate the effects of the PGE_2_ signaling under conditions in which arsenite promotes NADPH-dependent O_2_^−.^formation.

## Data Availability

The raw data supporting the conclusions of this manuscript will be made available by the authors, without undue reservation, to any qualified researcher.

## Author Contributions

OC conceived the research. LC, AG, and MF performed the experiments. LC, AG, and MF analyzed the data. OC wrote the manuscript. LC, AG, MF, and OC revised the manuscript. All authors approved the final version of the manuscript.

## Funding

This work was supported by Ministero dell’Università e della Ricerca Scientifica e Tecnologica, Programmi di Ricerca Scientifica di Rilevante Interesse Nazionale, 2015 (grant number 2015MJBEM2-003 to OC).

## Conflict of Interest Statement

The authors declare that the research was conducted in the absence of any commercial or financial relationships that could be construed as a potential conflict of interest.

## Abbreviations

ATZ, 3-amino-1,2,4,-triazole; cAMP, cyclic adenosine monophosphate; CsA, cyclosporin A; DHR, dihydrorhodamine 123; IBMX, 3-isobutyl-1-methylxanthine; MPT, mitochondrial permeability transition; mitoO_2_^−.^, mitochondrial O_2_^−.^; PGE_2_, prostaglandin E_2_; EP, E prostanoid receptor; PKA, protein kinase A; Ser^112^, serine 112; O_2_^−^, superoxide.
